# Effect of Comprehensive Rehabilitation Training Program in Orthopedic Nursing of Patients with Residual Limb Injury Caused by Crush

This article has been retracted.

**DOI:** 10.1155/2022/6769572

**Published:** 2022-01-25

**Authors:** Haihong Zhou, Tongyao Yu

**Affiliations:** ^1^Department of Hand and Foot Surgery, The First People's Hospital of Wenling, Wenling, Zhejiang 317500, China; ^2^Department of Orthopedic Trauma, The First People's Hospital of Wenling, Wenling, Zhejiang 317500, China

## Abstract

This study was developed to explore the role and application value of a comprehensive rehabilitation training (CRT) program based on the remote monitoring system of limb rehabilitation training (LRT-RM system) in the rehabilitation nursing of patients with residual limb injuries caused by crush. The LRT-RM system was constructed based on the characteristics of limb movement and using the time-domain analysis method and support vector machine (SVM). The 84 crush injury patients were selected as the research objects and divided into a control group (Con group, received conventional rehabilitation therapy) and a CRT group (received conventional rehabilitation therapy + functional training) according to different therapies, with 42 people in each group. The incidence of compound injuries and the incidence of residual limb injuries were counted and compared for patients in two groups. The differences in renal function, blood electrolytes, and biochemical indicators before and after treatment were analyzed. The MOS 36-item short-form health survey (SF-36) scale was selected to evaluate the improvement of physical and mental health of the patients before treatment and 1 month (time point (TP1)), 3 months (TP2), 6 months (TP3), and 12 months (TP4) after the treatment. It was found that, after the intervention, the values of serum creatinine (Scr), blood urea nitrogen (BUN), uric acid (UA), K^+^, P^3+^, and white blood cells (WBC) of patients in CRT group were obviously lower than those of Con group (*P* < 0.05), and the values of carbon dioxide combining power (CO_2_CP), Ca^2+^, hemoglobin (Hb), red blood cell (RBC), total protein (TP), and albumin (ALB) were obviously higher than the values in Con group (*P* < 0.05). In the CRT group, the residual limb injury rate was lower in elbow, wrist, shoulder joint, ankle joint, and toe (*P* < 0.05) and extremely lower in knee joint in contrast to that in the Con group (*P* < 0.001). The score of SF-36 was dramatically higher than that in the Con group (*P* < 0.05). It suggested that the CRT program based on the LRT-RM system was helpful for the rehabilitation of patients with crush injuries, and it can reduce the incidence of residual limb injuries in patients. Results of this study could provide a reference basis for the treatment of residual limb injuries caused by crush.

## 1. Introduction

Crush injury is caused by ischemia damage of the limbs and muscles being buried under heavy objects for a long time due to the destruction of traffic, water, electricity, and communication, as well as natural disasters such as earthquake and tsunami [1, 2]. In the later stage of residual limb injuries, varying degrees will affect the body's sensory or motor function and seriously affect the quality of life of patients [3, 4]. Reasonable comprehensive rehabilitation therapy (CRT) programs and surgical methods are often used for treatment, which has been proved in many studies [5]. CRT is an organic combination of multiple rehabilitation methods, which is mostly used in the treatment of mid-term crush injury [6]. Active CRT mainly includes functional training, psychotherapy, and physical therapy, and it aims to promote the recovery of limb function [7]. The limb swelling of patients will gradually disappear after 3 to 4 weeks after a crush injury. At this time, effective CRT therapy can greatly improve the function of the remaining muscles and prevent joint stiffness and muscle contracture [8]. At present, there are many researches on the early treatment of crush injury patients all over the world, but there are few studies on the rehabilitation treatment of residual limb injuries in the later period of crush injury.

Due to uneven distribution of domestic medical conditions and limited economic conditions, many patients cannot receive the effective rehabilitation guidance of professional rehabilitation doctors, which may prolong the recovery time and inhibit the disease better of patients. Therefore, remote limb rehabilitation training under the guidance of professional rehabilitation physicians is of great significance to the crush injury patients. The remote monitoring system of limb rehabilitation training (LRT-RM system) can provide rehabilitation physicians with real-time movement data of patients and provide a basis for rehabilitation physicians to set up effective training plans. According to some documents, the LRT-RM system is superior with the characteristics of low price and high convenience [9], so it has been applied in aspects and has been studied in many researches. Block et al. [10] designed a single-finger exoskeleton training device based on three-dimensional (3D) printing technology, but it shows some disadvantages such as poor flexibility and high cost. Qiu et al. [11] optimized the finger joint rehabilitation training device and initially realized remote rehabilitation, but it still showed the shortcomings of single system control and unstable performance, which has to be optimized further.

In summary, there are currently few domestic researches on the rehabilitation of residual limb injuries in the later stage of crush injury. At present, the LRT-RM system has to be further optimized so that it can meet the current requirements of practical use. Therefore, the LRT-RM system was constructed based on the characteristics of limb movement and using the time-domain analysis method and support vector machine (SVM), and the patients with crush injury were undertaken as the research objects receiving the CRT therapy to intervene, so as to analyze the application value of the LRT-RM system in the rehabilitation training of patients with crush injury and explore the rehabilitation effect of the CRT program based on the LRT-RM system on remaining injured limbs of patients with crush injury, aiming to provide the practical reference to treat the patients with crush injury.

## 2. Materials and Methods

### 2.1. Establishment of Recognition Method for Movement Signal of Limb Rehabilitation Training

The time-domain analysis method shows significant advantages to process the action signal waveform [12]. For a discrete signal {*x*_0_, *x*_1_, ⋯*x*_*n*_}, the discrete signal can be expressed as follows:

(1) $$\begin{array}{c} X=\frac{1}{n+1}\sum_{m=0}^{n}x_{m}. \end{array}$$

In the equation above, *n* is the number of discrete signals and *x*_*m*_ represents the *m*-th discrete signal.

Wavelet transform can analyze the signal from the perspective of time domain and frequency domain and can decompose the data signal at various levels, so that the extracted characteristic signal can be more accurate [13]. The continuous wavelet transform algorithm is given as follows:

(2) $$\begin{array}{c} \phi \left(t\right)=\frac{1}{\sqrt{a}}\phi \left(\frac{t-d}{a}\right), \end{array}$$

where *a* refers to the expansion factor, *t* refers to the time, and *d* is the translation factor.

The multiresolution analysis method decomposes and reconstructs the collected signal data to obtain high- and low-frequency component distribution signals, and the resolution of each segment is greatly different [14]. The multiresolution analysis method in wavelet transform can be expressed as in the following equation:

(3) $$\begin{array}{c} x\left(t\right)=\sum_{k=-\infty }^{\infty }a_{lk}\phi_{lk}\left(t\right)+\sum_{l=-\infty }^{\infty }\sum_{k=-\infty }^{\infty }g_{lk}\phi_{lk}\left(t\right). \end{array}$$

In the above equation, *ϕ*_*lk*_(*t*) refers to the scale function, ∑_*k*=−*∞*_^*∞*^*a*_*lk*_*ϕ*_*lk*_(*t*) shows the corresponding relationship in the representative space represented by *x*(*t*), *a*_*lk*_ represents the high-frequency component in the signal data, and *g*_*lk*_ is the low-frequency component in the signal data.

It is assumed that the collected signal is *B*, which can be expressed as in equation (4) after wavelet packet decomposition, where *i* is the number of decomposition layers and *n* represents the number of nodes.

(4) $$\begin{array}{c} B=B_{i,0}+B_{i,1}+\cdots +B_{i,\left(2^{n}-1\right)}. \end{array}$$

SVM classification method can realize intelligent classification and strong generalization, which can avoid machine overlearning [15]. In this study, the SVM classifier was adopted to analyze the data collected by the remote system. To analyze the training effect of the system, (*x*_1_, *y*_1_), ⋯, (*x*_*l*_, *y*_*l*_) (*x* ∈ *R* and *y* ∈ [−1,1]) were taken as the system training sample, and (*α·x*) − *β*=0 was set to the optimal classification surface, where *α* was the bias coefficient and *β* was the weight vector coefficient. According to the optimal hyperplane classification principle, the optimal classification hyperplane can be expressed as follows:

(5) $$\begin{array}{c} \left\{\begin{array}{cc} \left(\alpha \cdot x\right)-\beta \geq 1, & y_{i}=1,\\ \left(\alpha \cdot x\right)-\beta \leq -1, & y_{i}=-1. \end{array}\right. \end{array}$$

The core of classifier construction is to select the correct kernel function. The Radial Basis Function (RBF) kernel can project nonlinear matters into high-latitude space and then establish linear functions to solve nonlinear issues [16]. The calculation method of the RBF kernel is shown in equation (6), where *γ* represents the distance of the horizontal axis:

(6) $$\begin{array}{c} F\left(x_{i},x_{j}\right)=\exp\left(-\frac{{\left\|x_{i}-x_{j}\right\|}^{2}}{2\sigma^{2}}\right)=\exp\left[-\gamma {\left\|x_{i}-x_{j}\right\|}^{2}\right]. \end{array}$$

The information sensor is worn by the rehabilitation trainer to receive the different signal data generated by the movement, the wavelet transform filter is used to filter the interference signal, and the wavelet packet decomposition method is used to decompose the data signal to obtain the characteristic value of the data signal. The SVM classifier can further distinguish the signals, and the specific process of physical rehabilitation training action signal recognition is shown in Figure 1.

### 2.2. LRT-RM System

The subjects were required to wear the motion information collector (Bosch) to collect the data of different motions, and the obtained signal data were transmitted to the personal computer through the wireless transmission module after the wavelet preliminary filtering process. The feature vector of the exercise energy was calculated, and the data was classified through the SVM classifier and transmitted to the rehabilitation doctor through the network. The process of LRT-RM system is shown in Figure 2.

The three-axis accelerometer (Bosch) was adopted to detect the acceleration of rehabilitation training personnel.

### 2.3. Research Objects and Their Grouping

A total of 84 patients with crush injuries from January 2019 to March 2021 were selected as the research objects. The included research objects all received the rehabilitation treatment based on the remote monitoring system of the rehabilitation department of our hospital under the guidance of rehabilitation experts. Among them, there were 65 males and 19 females, and the age range was 21–68 years (with the average age of 38.24 ± 9.67 years). All cases met the diagnostic criteria for crush injury [17]. All study objects were divided into a control group (Con group, received conventional rehabilitation therapy) and a CRT group (received conventional rehabilitation therapy + functional training) according to different therapies, with 42 people in each group. The inclusion criteria of this study were defined as follows: patients who were diagnosed as crush injury; patients without acute renal failure and severe medical diseases; patients with normal consciousness; patients without obvious abnormalities of heart, brain, liver, lung, kidney, and blood coagulation in routine examinations; and patients who actively cooperated with doctors for examination and treatment, complete clinical diagnosis, treatment, and follow-up. The exclusion criteria were defined as follows: those who were unconscious and unable to cooperate; those with abnormal heart, brain, liver, lung, kidney, and blood coagulation functions; and those with immunosuppressive diseases, malignant tumors, and hematological diseases. The trial process of this study had been approved by the ethics committee of the hospital, and all subjects included in the study had signed the informed consent forms.

### 2.4. Nursing Interventions Programs

Patients in Con group were treated with conventional rehabilitation therapy. After one month, the symptoms and signs of patients did not improve obviously, and the walking or running function was severely affected. According to the nature and location of the damaged tissue, the corresponding surgical intervention was used for treatment [18]. Conventional rehabilitation therapy was based on the principles of dissipating indurations, softening scars, loosening adhesions and contractures, and improving local blood circulation. Nonsurgical wounds were treated with shortwave, ultrasound, or paraffin wax, with 15 min/time/day. Surgery patients were treated with shortwave or ultrasound within 15 days after surgery. Prostheses and corresponding orthoses were used for auxiliary intervention in different injured parts, and it can be combined with the electric acupuncture and massage methods of traditional Chinese medicine (TCM). Based on the actual dysfunction site and treatment operations of patients, the appropriate technique was used for massage, with 30 min/time and 2 times/day. It could refer to the method in the work of Fei et al. [19], which was mainly based on local acupoint selection and acupoint selection along the meridian, and the acupuncture treatment was performed with 15 min/time, 1 time/day, 10 times/course. The content of conventional rehabilitation therapy in the Con group is shown in Figure 3.

Patients in CRT group accepted CRT program. It provided appropriate functional training rehabilitation methods based on the conventional rehabilitation therapy. Different exercise therapies were selected to intervene according to different damaged parts, natures, and surgical methods. Joint movement was required 30 minutes each time with 2 times a day. According to the method of Geary et al. [20], the joint loosening technique was divided into 4 levels, and different techniques were used for intervention, each with 30 min/time and 2 times a day. The joint range of motion training and muscle strength training was performed for the injured part of nonsurgically wounded, with 30 min/time and 2 times/day; and for the wounded with tendon loosening, the toe flexion and extension activities were required 36 hours after the surgery. For patients with prolonged tendons, the calf triceps contraction exercise should be started on the 1st day after surgery, and then active toe flexion and extension exercises should be started 3 weeks later. For patients with distal tendon transection, the ankle and knee flexion and extension exercises were performed 3 days after the surgery.

### 2.5. Observation Indicators and Follow-Up

Basic data of the two groups of patients were recorded, such as age, gender, squeezed time, number of affected limbs, and past medical history. The proportions of compression parts and patients caused by different compression factors, compound injuries, and residual limb injuries of patients were calculated and compared. The differences in renal function, blood electrolytes, and biochemical indicators between the two groups of patients before and after treatment were analyzed and compared. The follow-up was continued for 1 year. The MOS 36-item short-form health survey (SF-36) scale was to evaluate the improvement of physical and mental health of patients before treatment and 1 month (time point (TP1)), 3 months (TP2), 6 months (TP3), and 12 months (TP4) after treatment.

### 2.6. Statistical Analysis

The data was processed using SPSS 19.0. The mean ± standard deviation ($\bar{x}$ ±  *s*) was to express the measurement data (*t*-test), and percentage (%) was to express the count data (*χ*^2^ test). *P* < 0.05 indicated that the difference was statistically significant.

## 3. Results and Discussion

### 3.1. Analysis on Data Collected by LRT-RM System

As given in Figure 4, the LRT-RM system collected different accelerations in different directions of the subjects. The fluctuations in the *X*-axis direction were the most severe, and the *Y*-axis and *Z*-axis data showed obvious periodicity, indicating that the acceleration value changes in the *X*-axis direction were the most obvious. The *Y*-axis data reflected the number of actions of the trainer, and the *Z*-axis data can determine whether the trainer had a turning action. During the limb training, the waveform signal of the trainer's limbs would fluctuate when the limbs were turning; otherwise, it would be in a stable state.

### 3.2. Comparison on Clinical Data of Patients

Statistics and analysis results of age, gender ratio, squeezed time, and past medical history of patients in Con group and CRT group (Table 1) were not statistically different (*P* > 0.05).

### 3.3. Comparison on Compression Parts and Compression Factors

The proportions of patients under different limb compression factors in the two groups were compared, and the results are given in Figure 5. No obvious difference was found in the percentages of patients with crush injuries caused by compression factors of landslides, car accidents, cement boards, wooden boards, and bricks (*P* > 0.05).

Further comparison on the proportions of patients with different compression parts in the two groups (Table 2) showed no statistical difference for patients (*P* > 0.05).

### 3.4. Comparison on Biochemical Indicators before and after Intervention

The changes of renal function indicators were compared before and after the intervention, including serum creatinine (Scr), blood urea nitrogen (BUN), carbon dioxide combining power (CO_2_CP), and uric acid (UA), as illustrated in Figure 6. There was no remarkable difference in the renal function indicators of the patients before the intervention (*P* > 0.05). The Scr, BUN, and UA of the two groups of patients after the intervention were obviously decreased, which were statistically different (*P* < 0.05); the CO_2_CP of the both groups was increased greatly (*P* < 0.05); the Scr, BUN, and UA values of the CRT group were decreased observably, and the CO_2_CP was elevated (*P* < 0.05). The Scr and BUN values of patients with crush injury were obviously increased [21, 22], and the Scr and BUN values of patients were greatly decreased after different interventions, indicating that the metabolic acidosis of patients has been alleviated.

The K^+^, Ca^2+^, and P^3+^ concentrations in blood electrolytes of patients are compared in Figure 7. Before application of the therapy, there was no visible difference in the average K^+^, Ca^2+^, and P^3+^ concentrations between the two groups (*P* > 0.05). After the intervention of different rehabilitation methods, K^+^ and P^3+^ were greatly reduced (*P* < 0.05), while Ca^2+^ was obviously increased (*P* < 0.05); the K^+^, Ca^2+^, and P^3+^ concentrations of the Con group were 5.03 ± 0.57 mmol/L, 1.91 ± 0.16 mmol/L, and 2.85 ± 0.30 mmol/L, while those in CRT group were 4.43 ± 0.49 mmol/L, 2.51 ± 0.22 mmol/L, and 2.31 ± 0.18 mmol/L, respectively. The K^+^, Ca^2+^, and P^3+^ concentrations were remarkably different after intervention (*P* < 0.05). The K^+^ and P^3+^ concentrations of patients with crush injury are elevated, with hypocalcemia in the early stage and hypercalcemia in the later stage. After different interventions, the blood electrolytes of patients have changed, which effectively better the balance states of electrolytes and acid-base levels, showing obvious elevation in the CRT group.

The biochemical indicators before and after nursing were further compared with white blood cell count (WBC), red blood cell count (Hb), total red blood cell (RBC), total protein (TP), and serum albumin (ALB) (Figure 8). No obvious difference was found in the average values of WBC, Hb, RBC, TP, and ALB before nursing (*P* > 0.05). After the intervention of different rehabilitation methods, the WBC values were decreased greatly in both groups (*P* < 0.05), while the values of Hb, RBC, TP, and ALB were obviously higher (*P* < 0.05). In addition, there were great differences in the WBC, Hb, RBC, TP, and ALB values between different groups after intervention (*P* < 0.05).

### 3.5. Comparison on Incidence of Residual Limb Injuries

Figure 9 shows the statistical results for the incidence of residual limb injuries in different parts after intervention. The incidence of residual limb injuries in elbow, wrist, and hand in CRT group was lower (*P* < 0.05), that in shoulder joint, ankle joint, and toe was greatly lower (*P* < 0.01), and that in the knee joint was extremely lower (*P* < 0.001). The limbs of patients with crush injury suffer from soft tissue necrosis due to prolonged compression [23]. Due to the influence of various factors, even if effective treatment is used, it is still possible to form scars of muscles and nerves, which will cause the existence of residual limb injuries [24]. The incidence of residual limb injuries after CRT intervention was decreased dramatically, indicating that CRT program can effectively reduce the incidence of residual limb injuries in patients with crush injuries. The reason is that the running training in the Con group is increased, and the squeezing patients can stimulate the excitement of the injured muscle through training and shorten the time of the injured nerve [25]. On the other hand, training can effectively improve the internal environment of the nerve injury site, maintain joint mobility, enhance nerve conduction capacity, and then better the residual limb injuries of patients [26].

### 3.6. Comparison on the SF-36 Score

The SF-36 scores were compared before nursing and at TPs 1, 2, 3, and 4 after nursing (as revealed in Figure 10). The difference was not visible in the SF-36 scores before intervention (*P* > 0.05). The patient in CRT group showed higher SF-36 score (*P* < 0.05), obviously higher score (*P* < 0.01), and extremely obviously higher score (*P* < 0.001) at TP2, TP3, and TP4, respectively. It suggests that CRT program can improve the physical and mental health of patients effectively.

## 4. Conclusion

The LRT-RM system was constructed based on the characteristics of limb movement and the crush patients were taken as the objects to discuss the role of the CRT program based on the LRT-RM system in the rehabilitation of crush patients and its application value in nursing of residual limb injuries. It was found that the CRT program based on the LRT-RM system helped patients with crush injuries recover and reduced the incidence of residual limb injuries in crush patients. In addition, the CRT program based on the LRT-RM system provided a reference basis for the treatment of residual limb injuries for patients with crush injury. However, there were some shortcomings for this study. It only compared the incidence of residual limb injuries after intervention and did not count the coexisting symptoms of patients during the follow-up period, so the long-term effects of the CRT program could not be evaluated. In future work, the complications and tissue repair status of patients during the follow-up period will be evaluated. In short, the CRT program based on the LRT-RM system provided a reference basis for the treatment of residual limb injuries for patients with crush injury.

## Figures and Tables

**Figure 1:** Flowchart of motion signal recognition for limb rehabilitation training.

**Figure 2:** Flowchart of LRT-RM system.

**Figure 3:** The content of conventional rehabilitation therapy.

**Figure 4:** Training data detected by the LRT-RM system.

**Figure 5:** Comparison on the proportion of patients under different limb compression factors.

**Figure 6:** The changes of renal function indicators. *Note.*^*∗*^ means *P* < 0.05 for the values before intervention; # means *P* < 0.05 for the Con group.

**Figure 7:** Comparison on blood electrolytes parameters. *Note.*^*∗*^ means *P* < 0.05 for the values before intervention; # means *P* < 0.05 for the Con group.

**Figure 8:** Comparison on biochemical indicators. (a) Comparison of WBC and RBC values of the two groups of patients before and after treatment; (b) comparison of Hb, TP, and ALB values of the two groups of patients before and after treatment. Note: ^*∗*^ means *P* < 0.05 for the values before intervention; # means *P* < 0.05 for the Con group.

**Figure 9:** Comparison on incidence of residual limb injuries. ^*∗*^, ^*∗∗*^, and ^*∗∗∗*^ suggest that the difference is obvious (*P* < 0.05), very obvious (*P* < 0.01), and extremely obvious (*P* < 0.001) in contrast to Con group, respectively.

**Figure 10:** Comparison on the SF-36 score. ^*∗*^, ^*∗∗*^, and ^*∗∗∗*^ suggest that the difference is obvious (*P* < 0.05), very obvious (*P* < 0.01), and extremely obvious (*P* < 0.001) in contrast to the Con group, respectively.

**Table 1:** Comparison on basic data of patients.

	Con group (*n* = 42)	CRT group (*n* = 42)	*t* value or *χ*^2^ value	*P* value
Age (years old)	37.92 ± 8.64	38.45 ± 9.13	1.764	0.223
Males (cases, (%))	33 (78.57%)	32 (76.19%)	2.254	0.285
Females (cases, (%))	9 (21.43%)	10 (23.81%)	0.068	0.791
Compression duration (h)	1.25 ± 0.42	1.28 ± 0.39	0.211	0.892

Past history of chronic disease				
Open injury	5 (11.90%)	6 (14.29%)	0.273	0.864
Closed injury	14 (33.33%)	13 (30.95%)		

**Table 2:** Distribution on patients with different compression parts.

Compression parts	Con group (*n* = 42)	CRT group (*n* = 42)	*χ* ^2^ value	*P* value
Left upper limb (cases, (%))	5 (11.90%)	6 (14.29%)	0.066	0.719
Right upper limb (cases, (%))	10 (23.81%)	11 (26.19%)	0.522	0.482
Both upper limbs (cases, (%))	4 (9.52%)	3 (7.14%)	0.183	0.785
Left lower limb (cases, (%))	5 (11.90%)	6 (14.29%)	0.242	0.894
Right lower limb (cases, (%))	8 (19.05%)	7 (16.67%)	0.054	0.662
Both lower limbs (cases, (%))	5 (11.90%)	4 (9.52%)	0.198	0.916
Left upper and lower limbs (cases, (%))	1 (2.38%)	1 (2.38%)	0.227	0.883
Right upper and lower limbs (cases, (%))	3 (7.14%)	3 (7.14%)	0.143	0.825
Limbs (cases, (%))	1 (2.38%)	1 (2.38%)	0.482	0.491

## Data Availability

The data underlying the results presented in the study are available within the manuscript.
